The article "Postoperative Cognitive Behavioral Intervention in Patients with Coronary Heart Disease Based on the Effect of Nursing Process Reengineering" was retracted in 2023. Reasons: signs of a paper mill; suspected computer-generated content; unreliable results or conclusions; lack of ethics approval or compliance.

# Postoperative Cognitive Behavioral Intervention in Patients with Coronary Heart Disease Based on the Effect of Nursing Process Reengineering

**DOI:** 10.1155/2022/6974909

**Published:** 2022-09-17

**Authors:** Ying Xiong, Yan Liu, Jianying Cui

**Affiliations:** ^1^Department of Cardiology, People's Hospital of Xinjiang Uygur Autonomous Region, Urumqi, 830001 Xinjiang, China; ^2^Department of Neurology, People's Hospital of Xinjiang Uygur Autonomous Region, Urumqi, 830001 Xinjiang, China; ^3^Department of Cadre Health Center, People's Hospital of Xinjiang Uygur Autonomous Region, Urumqi, 830001 Xinjiang, China

## Abstract

With the development of society and economy, patients with coronary heart disease increasingly hope to receive more humanized services after surgery, and the reengineering of the nursing process is precisely based on humanized management. In order to create a nursing intervention that helps in boosting total nursing gains and lowering disasters, the primary element of the nursing business process reengineering is to reintegrate or condense the creative work flow that was fragmented by specialization into a whole job. The “patient” is positioned in the center of nursing process reengineering, with service quality as the main guiding principle. It follows the management principles of continuous regulation and innovation, and cultivates and promotes the development of the nursing field from the perspective of “sublation.” In the method part, this article introduces and supplements related information on nursing process reengineering, coronary heart disease, and postoperative cognitive behavioral intervention. Algorithmically, this paper proposes 3D RPN structure, loss function, capsule network, and improved activation function algorithm for coronary heart disease region extraction. In the part of experiment and results, this article collects general data of patients and compares memory ability, grades of self-management behaviors of patients treated with coronary heart disease, scores of quality control standards before and after nursing process reengineering, scores of patients' mental state, and comparison of postoperative physical indicators. According to the test results, the test group's diastolic and systolic blood pressure declined by more than 20, their total cholesterol dropped from 6.23 to 5.28, and their triglyceride levels dropped from 1.82 to 1.39 after the stent was implanted. Triglycerides reduced from 1.82 to 1.39, and total cholesterol dropped from 6.15 to 5.98. It indicates postoperative memory in patients with coronary heart disease. Abilities, including recognition, number, touch memory, and associative memory, decline significantly, but it can be improved after receiving the nursing process reengineering. It can be seen that nursing process reengineering can play a positive role in the postoperative cognitive behavior of patients with coronary heart disease.

The article "Postoperative Cognitive Behavioral Intervention in Patients with Coronary Heart Disease Based on the Effect of Nursing Process Reengineering" was retracted in 2023. Reasons: signs of a paper mill; suspected computer-generated content; unreliable results or conclusions; lack of ethics approval or compliance.

## 1. Introduction

Postoperative cognitive dysfunction refers to the complications of the central nervous system that often occur after surgery, manifested as mild confusion and tendency to fantasies, memory forgetting, inner restlessness or unfounded fear, and personality, social skills, and cognition changes in abilities and skills; POCD mostly appear in the early postoperative period to several months after surgery and may last for a long time. POCD seriously affects the quality of life of patients, prolongs the length of hospitalization, increases hospitalization costs, affects the prognosis of the disease, and even develops into senile dementia. The etiology of POCD is not yet clear, the triggers are many, the clinical manifestations are complicated, and it is difficult to distinguish from postoperative delirium. The treatment methods have not yet unified standards. They are often ignored by medical staff and cannot be diagnosed in time, which makes it impossible to give timely diagnosis. Effective intervention therapy has become the focus of perioperative medicine.

Based on the effect of nursing process reengineering on postoperative cognitive behavioral intervention in patients with coronary heart disease, many scholars at home and abroad have conducted related research. Konrad et al. determined the prevalence and risk factors of depression in patients. The main outcome measure is the initial diagnosis of depression in patients with and without CHD within five years of the index date. The Cox proportional hazard model is used to adjust for confounding factors [1]. Lindgreen et al. believe that patients who undergo lumbar fusion surgery are generally assisted, which is considered an effective intervention to improve beneficial pain-coping behaviors and thus facilitate the recovery process for patients with chronic pain. The recipient prevents or minimizes pain by resting before the onset of pain, while the nonrecipient waits for the onset of pain before resting. The postoperative experience brings ambivalence, causing uncertainty, worry, and insecurity. When others recognize the patient's pain and provide support, this ambivalence is relieved. As part of rehabilitation, cognitive behavioral therapy may encourage beneficial pain-coping behaviors. The author conducted related research on postoperative intervention but did not propose a specific solution [2]. Müller-Staub et al. proposed that nurses are responsible for applying the nursing process, which is essential for patient care: It is a problem-solving process that provides structure for nursing plans and documentation. The author sorted out the nursing process but only conducted an interview study on the nursing process, without combining specific data [3].

The article "Postoperative Cognitive Behavioral Intervention in Patients with Coronary Heart Disease Based on the Effect of Nursing Process Reengineering" was retracted in 2023. Reasons: signs of a paper mill; suspected computer-generated content; unreliable results or conclusions; lack of ethics approval or compliance.

In this paper, based on the nursing process reengineering, the method of postoperative cognitive behavior intervention in patients with coronary heart disease was studied. In the method part, this article introduces and supplements related information on nursing process reengineering, coronary heart disease, and postoperative cognitive behavioral intervention. Algorithmically, this paper proposes 3D RPN structure, loss function, capsule network, and improved activation function algorithm for coronary heart disease region extraction. In the part of experiment and results, this article collects general data of patients and compares memory ability, grades of self-management behaviors of patients treated with coronary heart disease, scores of quality control standards before and after nursing process reengineering, scores of patients' mental state, and comparison of postoperative physical indicators. The innovation of this article is to use nursing process reengineering to improve the cognitive behavior of patients with coronary heart disease after surgery and to conduct scientific interventions on these behaviors to help patients achieve good postoperative recovery.

## 2. Postoperative Cognitive Behavioral Intervention Method in Patients with Coronary Heart Disease Based on the Effect of Nursing Process Reengineering

### 2.1. Nursing Process Reengineering

Nursing business process reengineering is to reengineer the weak, hidden danger and unrealistic links of the original nursing work process, through the integration, deletion, reorganization and reconstruction of the original business process, and the reconstructed work process. The nursing process increases the proportion of nurses' work in the overall emergency process and not only makes full use of nurses' mobility, reduces the high burden of emergency doctors, and reduces the cost of human resources but also improves nurses' sense of professional honor [4, 5]. Nursing has long become a first-level discipline as important as clinical. Nurses should not only be doctors' assistants. Increasing the proportion of work and improving their own abilities are one of the manifestations of nurses' professional value [6].  Figure 1 shows the nursing process reengineering model.

Members of the rehabilitation process are the vice president of the hospital, the director of the nursing home, the head of the emergency department, the head of the cardiology department, the head of the cardiovascular center, the emergency physicians, the emergency nurses, and other emergency personnel [7]. Among them, the vice president of the hospital, as the reengineering organizer, is responsible for the overall planning and decision-making of the entire research process; the director of the nursing department and the head nurse of the emergency department and the cardiology department have rich management and clinical experience and can provide strong support for process analysis and reorganization. As the backbone of the reengineering process, the person in charge of the Coronary Heart Disease Center is familiar with related content such as the operation process and evaluation indicators of the Coronary Heart Disease Center, which is an important support for research. The establishment of an emergency care process based on the Coronary Heart Disease Center further enhances its scalability: emergency doctors [8, 9].  Figure 2 shows the emergency node diagram.

The article "Postoperative Cognitive Behavioral Intervention in Patients with Coronary Heart Disease Based on the Effect of Nursing Process Reengineering" was retracted in 2023. Reasons: signs of a paper mill; suspected computer-generated content; unreliable results or conclusions; lack of ethics approval or compliance.

### 2.2. Coronary Heart Disease

Atherosclerotic coronary heart disease is caused by coronary atherosclerosis, which causes vascular stenosis, blockage, or spasm, causing myocardial ischemia, hypoxia, or necrosis, also referred to as coronary heart disease [10]. It includes five types of treatment: angina, myocardial infarction, asymptomatic myocardial ischemia (coronary heart disease), ischemic heart failure, and sudden death, which can cause palpitations, fatigue, other heart attacks, and depression. [11, 12].

As the most common and frequent cardiovascular disease, it accounts for 67.1% of the mortality rate of cardiovascular diseases. Coronary heart disease has the characteristics of complex pathogenesis, high morbidity, high recurrence rate, high mortality, and expensive medical expenses. It is the world's disability and one of the main causes of death [13]. The World Health Organization said that in the next ten years of development, the danger of cardiovascular disease will continue to rise. It is estimated that by 2030, the mortality rate of coronary heart disease patients will account for 13.1% of the total population of coronary heart disease. With the acceleration of the aging of our country's population, the incidence of coronary heart disease is getting younger and younger, and the mortality rate of coronary heart disease is gradually increasing.  Figure 3 shows the symptoms and treatment of coronary heart disease.

The incidence of coronary heart disease is related to the following factors: (1) age: In recent years, surveys have shown that the population of coronary heart disease is still dominated by the elderly, but the proportion of age is decreasing year by year; the proportion of middle-aged and young patients is increasing year by year. (2) Gender: The incidence of men is higher than that of women, and there are surveys that the risk of severe coronary heart disease (coronary artery stenosis ≥75%) in women is only half that of men, but the incidence of women after menopause has begun to rise, which may be related to the decline in hormone levels. (3) Others: The currently recognized risk factors for coronary heart disease include hypertension, hyperlipidemia, diabetes, obesity, genetics, smoking, and so on. The content of coronary heart disease-related knowledge is divided into eight dimensions: coronary heart disease-related concepts, risk factors, predisposing factors, clinical manifestations, examination items, treatment methods, drug knowledge, secondary prevention, and total coronary heart disease knowledge. The results showed that after the intervention, the scores and total scores of the two groups of patients' coronary heart disease-related knowledge were improved compared with before the intervention, indicating that both in-hospital routine nursing and information-based continuous nursing can improve the level of coronary heart disease-related knowledge. At 3 months and 6 months after discharge, the scores and total scores of all dimensions of coronary heart disease-related knowledge in the intervention group were higher than those in the control group, and the scores were significantly different (*P* < 0.05), indicating that the information-based continuous nursing intervention model is better [14, 15]. The reasons are as follows: ① The information-based continuous nursing intervention model continues to provide patients with correct health guidance, ensures the continuity of the treatment relationship, and enhances the patient's determination to defeat the disease. ② The information-based continuous nursing intervention model is guided by nurses, and multidisciplinary personnel participate and cooperate to complete it and implement a planned, focused, hierarchical, staged, and diverse form of professional and information-based nursing intervention model to replace the traditional cramming education. They pay attention to not only the physical health of the patients but also the psychological health and emotional stability of the patients and promote the patients to establish a good and positive attitude to deal with the disease. ③ Under the informatization continuation care model, the intervener implements individualized guidance to the patient and performs phased interventions according to the actual situation of the patient, so that patients get mutual encouragement and support from peers and urge each other to persevere better [16, 17].  Figure 4 is an electrocardiogram and obstruction of coronary heart disease.

The article "Postoperative Cognitive Behavioral Intervention in Patients with Coronary Heart Disease Based on the Effect of Nursing Process Reengineering" was retracted in 2023. Reasons: signs of a paper mill; suspected computer-generated content; unreliable results or conclusions; lack of ethics approval or compliance.

### 2.3. Cognitive Behavior of Patients after Surgery

Currently, therapeutic practice frequently uses cognitive behavioral interventions as psychological interventions. It is a methodical kind of psychotherapy. Yes, cognitive behavioral intervention holds that behavioral and cognitive processes may interact and affect one another. This intervention technique primarily alters the patient's irrational cognition through technological correction and the combined correction of cognition and behavior. In order to help patients rebuild their understanding of cognitive behavioral treatment methods, therapeutic learning classes, systematic teaching of treatment theories, and one-on-one conversations are typically used. Patients are also given examples of appropriate responses, system desensitization, relaxation training, etc., to help them relieve the burden.

The cause of postoperative cognitive dysfunction is not yet clear; there are many triggers; the clinical manifestations are complex, and it is difficult to distinguish from postoperative delirium. The treatment methods have no unified standards, and they are often ignored by medical staff and cannot be diagnosed in time, resulting in failure. Early and timely and effective intervention treatment has become the focus of perioperative medicine [18]. The compensatory ability of the patient's body gradually degrades with the age of the patient, which has led to a gradual increase in the prevalence of POCD in patients, and even the prevalence of POCD in the population >65 years old is 2–10 times that of the population <65 years old, which has caused society.

Cognitive behavioral intervention is a technique used to study the thinking and behavior of individuals and to help people solve bad mental states and behavioral problems. Cognition includes automatic thinking and beliefs. Its changes need to be corrected with therapeutic guidance techniques. Psychologists believe that individual cognition affects the production and development of mental states and behaviors, and at the same time, cognition will be affected by mental states and behavior [19]. This kind of cognitive behavioral intervention is to use some methods and techniques to help patients judge whether the response to an event is appropriate, test whether the patient's understanding of things is appropriate and the reasons for the bad mental state and behavior, and use the surrounding resources to deal with it, so as to gradually change the patients' bad cognition, mental state, and behavior; establish a virtuous circle between the three; and then improve the bad psychology and behavior. Its commonly used general strategies are cognitive reconstruction, behavior modification, relaxation training, acceptance, etc. Many studies have proved its uniqueness and importance in intervention, which can improve clinical efficacy, reduce negative emotions, increase confidence in overcoming diseases, and improve quality of life [20]. The advantage of this intervention method is that it has a strong theoretical tolerance; the intervention treatment has a wide range of treatments, and the causes of psychological problems are more complicated. An outstanding problem may be a combination of multiple problems. Therefore, the breadth of the treatment method is a standard to measure.

The article "Postoperative Cognitive Behavioral Intervention in Patients with Coronary Heart Disease Based on the Effect of Nursing Process Reengineering" was retracted in 2023. Reasons: signs of a paper mill; suspected computer-generated content; unreliable results or conclusions; lack of ethics approval or compliance.

The principles of cognitive behavioral intervention are as follows: (1) It requires cooperation between medical staff and patients and emphasizes the enthusiasm of participation. (2) The educational effect of cognitive behavioral intervention is embodied in that it aims at patients' self-management. (3) Cognition plays an intermediary and coordinating role in mental state and behavior. An individual's views and feelings about an event are the direct cause of a certain mental state and behavior when an individual is faced with an event. Mental state will in turn affect the individual's cognition. (4) The premise of cognitive behavioral intervention is to tap the patient's understanding and knowledge of things and behaviors. (5) Cognitive behavioral intervention is goal-oriented, focusing on solving the patients' current problems. In this intervention, the patient is an active individual, and the treatment effect depends on the patient's active participation. The patient should and has the responsibility to be responsible for his body and psychology.

### 2.4. Extraction of Coronary Heart Disease Area

#### 2.4.1. 3D RPN Structure

In faster RCNN, the RPN was first proposed to replace the selective search algorithm to generate candidate boxes. This network shares the backbone network for feature extraction with the RCNN, and the feature extraction network, RPN, and RCNN are trained at the same time. The detection algorithm realizes the end-to-end training and testing of the target detection task.

Among the methods to deepen the convolutional neural network longitudinally, the most typical one is the VGG network structure, which deepens the overall network by stacking convolutional layers. But when the depth of the network reaches a certain level, even in the case of batch normalization, the network of the VGG structure is difficult to converge, because the deep gradient will disappear when the deep gradient is backpropagated. The residual network solves this problem very well, so that the network can be deepened to a few hundred or even a thousand layers in the vertical direction. Let *m* be the input and *g*(*m*) be the output of the network in the residual unit, and the final output can be expressed as the following formula:

(1) $$\begin{array}{c} V\left(m\right)=g\left(m\right)+m, \end{array}$$

where *V*(*m*) is the final output of the network structure, because the input *m* is known; then, what the network structure actually learns is

(2) $$\begin{array}{c} g\left(m\right)=V\left(m\right)-m. \end{array}$$

The article "Postoperative Cognitive Behavioral Intervention in Patients with Coronary Heart Disease Based on the Effect of Nursing Process Reengineering" was retracted in 2023. Reasons: signs of a paper mill; suspected computer-generated content; unreliable results or conclusions; lack of ethics approval or compliance.

#### 2.4.2. 3D RPN Loss Function

There are three tasks in the 3D RPN, which are to determine the coordinates of coronary heart disease, predict the diameter of the heart, and identify all samples belonging to lung nodules in the anchor. The coordinates and diameters of the lung nodules are predicted to belong to the regression task, and the mean square error (*K*_2_ loss) or square absolute error (*K*_1_ loss) is used to optimize these two tasks, while identifying lung nodules in anchors belongs to the classification task, and the cross-entropy loss function can be used to optimize this task.

When the input is *m*, the real label is *N*, and the operation of the network is simply expressed as a function *g*; then, the output is *g*(*m*). Then, the *K*_2_ loss has the following calculation relationship and derivative:

(3) $$\begin{array}{c} K_{2}\left(m\right)={\left|g\left(m\right)-N\right|}^{2},\\ K_{2}^{\prime }=\left(m\right)2\left(g\left(m\right)-N\right)f^{\prime }\left(m\right). \end{array}$$

*K*_1_ loss and its derivative can be calculated according to the following formula:

(4) $$\begin{array}{c} K_{1}\left(m\right)={\left|g\left(m\right)-N\right|}^{2},\\ K_{1}^{\prime }\left(m\right)=\pm g\left(m\right). \end{array}$$

It can be found that the gradient of the *K*_1_ loss function is only related to the input value, and the difference between the predicted value and the target value is not well reflected on the gradient. Considering the above situations, this article adopts a new loss function called smooth *K*_1_ loss, which can be calculated by the following formula:

(5) $$\begin{array}{c} {\text{smooth}}_{K1}\left(n\right)=\left\{\begin{array}{cc} 0.5n^{2} & \left|n\right|<1\\ \left|n\right|-0.5 & \text{otherwise} \end{array}\right., \end{array}$$

where *y* is the error between the predicted value and the target value:

(6) $$\begin{array}{c} n=g\left(m\right)-N. \end{array}$$

When the total sample size is *P*, *l*_*x*_ and ln_*x*_, respectively, represent the predicted value and true value of the diameter of the *x*th sample, and *b*_*xy*_ and *bn*_*xy*_, respectively, represent the predicted value and true value of the coordinate of the *x*th sample, where *y* represents the *y*th coordinate of the sample, There are three types of *m*, *n*, and *q* in total, so the final position loss and size loss can be calculated separately by the following formulas:

(7) $$\begin{array}{c} K_{\text{loc}}\left(l,\ln\right)=\overset{J}{\underset{x}{\sum }}\left|l_{x}=1\right|{\text{smooth}}_{K_{1}}\left(l_{x},\ln_{x}\right),\\ K_{\text{coord}}\left(b,bn\right)=\overset{J}{\underset{x}{\sum }}\overset{3}{\underset{y}{\sum }}\left|b_{x}=1\right|{\text{smooth}}_{K_{1}}\left|\left(l_{xy},\ln_{xy}\right)\right.. \end{array}$$

Assuming that *r*_*x*_ and *N*_*x*_, respectively, represent the predicted value and true value of the *x*th difficult sample, then the loss function of the classification network can be calculated by the following formula:

(8) $$\begin{array}{c} K_{clc}\left(r,N\right)=\overset{t}{\underset{x}{\sum }}N_{x}\log\left(r_{x}\right)+\left(1-Y_{x}\right)\log\left(1-r_{x}\right). \end{array}$$

The loss function of 3D RPN is:

(9) $$\begin{array}{c} K_{rpn}=K_{loc}+K_{coord}+K_{clc} \end{array}$$

The article "Postoperative Cognitive Behavioral Intervention in Patients with Coronary Heart Disease Based on the Effect of Nursing Process Reengineering" was retracted in 2023. Reasons: signs of a paper mill; suspected computer-generated content; unreliable results or conclusions; lack of ethics approval or compliance.

#### 2.4.3. Capsule Network

The parameters ${\hat{v}}_{y/x}$ and *t*_*y*_ are the weight parameters of intermediate vectors *Q*_*xy*_ and *b*_*xy*_, which represent the output, and squashing represents the activation function.

(10) $$\begin{array}{c} {\hat{v}}_{y/x}=Q_{xy}v_{x},\\ b_{xy}=\frac{\exp\left(a_{xy}\right)}{\sum_{r}\exp\left(a_{xr}\right)},\\ t_{y}=\underset{x}{\sum }b_{xy}{\hat{v}}_{y/x}. \end{array}$$

The activation function of the capsule network is as follows:

(11) $$\begin{array}{c} u_{y}=\frac{{\left\|t_{y}\right\|}^{2}}{1+{\left\|t_{y}\right\|}^{2}}\frac{t_{y}}{{\left\|t_{y}\right\|}^{2}}. \end{array}$$

#### 2.4.4. Improve the Activation Function

The activation function used by the capsule network is as follows:

(12) $$\begin{array}{c} u_{y}=\alpha \frac{t_{y}}{\left\|t_{y}\right\|}=\frac{{\left\|t_{y}\right\|}^{2}}{1+{\left\|t_{y}\right\|}^{2}}\frac{t_{y}}{{\left\|t_{y}\right\|}^{2}}. \end{array}$$

Among them, the coefficient *α* can be regarded as transformed from the following formula:

(13) $$\begin{array}{c} n=\frac{m^{2}}{1+m^{2}}. \end{array}$$

It is difficult to obtain an activation function in the capsule network, and the recognition accuracy of the capsule network is not very high. The new activation function and expression are proposed as follows:

(14) $$\begin{array}{c} n=\left(1-e^{-0.5m^{2}}\right),\\ u_{y}=\left(1-e^{-0.5{\left\|t_{y}\right\|}^{2}}\right)\frac{t_{y}}{\left\|t_{y}\right\|}. \end{array}$$

The article "Postoperative Cognitive Behavioral Intervention in Patients with Coronary Heart Disease Based on the Effect of Nursing Process Reengineering" was retracted in 2023. Reasons: signs of a paper mill; suspected computer-generated content; unreliable results or conclusions; lack of ethics approval or compliance.

## 3. Postoperative Cognitive Behavioral Intervention Experiment and Result in Patients with Coronary Heart Disease Based on the Effect of Nursing Process Reengineering

### 3.1. General Patient Data

A comparison of the general information of the two groups of patients is shown in Table 1. General personal data (age, gender, level of education, smoking, etc.) of the project team and the control group were compared, and hospital data related to the disease (dates of hospitalization, number of stent inserts, number of drugs, etc.) are compared. The results showed that there was no statistically significant difference in general information between the two groups of patients (*P* > 0.05), and the two groups of patients were balanced and comparable.

### 3.2. Comparison of Memory Ability

As shown in Figure 5, the scores of memory ability in T2 and T3 phases of the control group are lower than those of the same group at T1 phase. For the index of recognition, the index is 11.87 at T1, 6.12 at T2, and 9.09 at T3. The postoperative memory ability of patients with coronary heart disease is reduced, among which touch memory and associative memory are significantly reduced.

As shown in Figure 6, there was no significant difference in MAP and HR between the two groups of patients 2 days before surgery, during skin surgery, 2 hours during surgery, and at the end of surgery. The MAP and HR of group patients were significantly higher than those of group I (*P* < 0.05).

As shown in Figure 7, there was no statistically significant difference in VAS and PONV numbers between the two groups 1 and 2 days after surgery. The incidence of group C patients was slightly higher than that of group C and group I. The ground work time in group C is slightly longer than that of group I.

Figure 8 shows a comparison of the incidence of POCD between the two groups of patients. The timeframe is set at 3 days before surgery, 1 day after surgery, and 7 days after surgery. You can see that the incidence of POCD in group C was high 1 and 3 days after surgery in group I.

### 3.3. Classification of Self-Management Behaviors of Patients Treated with Coronary Heart Disease

The postoperative self-management of patients with coronary heart disease is shown in Figure 9. It can be seen that the proportion of patients with medium level is the largest, and patients with low level are slightly lower than those with medium level. The high-level patients are much lower than the other two, which shows that patients have a lack of knowledge after surgery and need to reengineer the nursing process.

### 3.4. Score of Quality Control Standards before and after Nursing Process Reengineering

Table 2 shows the indicators of the two groups of patients before and after the reconstruction, including basic nursing, hemodialysis knowledge, nursing operations, and other indicators. It can be seen that the quality before the reconstruction is significantly lower than that after the reconstruction.

The article "Postoperative Cognitive Behavioral Intervention in Patients with Coronary Heart Disease Based on the Effect of Nursing Process Reengineering" was retracted in 2023. Reasons: signs of a paper mill; suspected computer-generated content; unreliable results or conclusions; lack of ethics approval or compliance.

### 3.5. Patient Mental State Score

Table 3 shows the psychological status of the observation group of the experimental group and the control group, including symptoms such as somatization, depression, anxiety, communication sensitivity, and obsessive-compulsive disorder. Obviously, the psychological score of the experimental group is lower than that of the control group, *P* < 0.05; the difference is statistically significant.

### 3.6. Comparison of Postoperative Indicators

As shown in Figure 10, after the stent was implanted, the serum AFABP and IL-6 levels of patients with various coronary heart diseases were observed. The reduction after stent placement was the lowest in the AMI group, but there was no significant difference in AFABP and IL-6 between UAP patients and AMI patients after PCI.

Table 4 shows the changes in blood lipids and blood pressure of the experimental group and the control group. After stent implantation, the test group had diastolic and systolic blood pressure decreased by more than 20, total cholesterol decreased from 6.23 to 5.28, and triglyceride also decreased from 1.82 to 1.39. Total cholesterol decreased from 6.15 to 5.98, and triglyceride also decreased from 1.82 to 1.39. It can be seen that after the intervention, blood pressure and blood lipids were significantly reduced, and the degree of reduction in the experimental group was higher than that of the control group.

## 4. Discussion

People have gradually deepened their understanding of the relationship between psychosocial factors and coronary heart disease. Researchers continue to propose new psychological treatment methods and psychological nursing theories. Psychological intervention therapy is also more and more widely used in clinical tumor treatment. More and more studies have shown that cognitive behavioral therapy has a significant effect on reducing the various stress responses of patients with coronary heart disease, allowing patients to complete the operation in the best condition. Cognitive therapy is one of the most extensive psychotherapy methods in the field of psychotherapy. Due to its remarkable effects and strong operability, it has attracted more and more attention in recent years and has gradually been widely used in clinical psychology. Cognitive behavioral intervention therapy is currently a highly recognized psychotherapy method in the world. It has been slowly developed after decades of exploration and research. It is an emerging psychological nursing intervention after psychoanalytic therapy and behavioral therapy method. Studies have concluded that POCD patients often have anxiety symptoms such as restlessness, nervousness, insomnia, and restlessness, and anxiety is a manifestation of psychological stress. Elderly patients are mostly due to their weak psychological endurance, and they have difficulties in adapting to the unfamiliar environment such as the disease, ward, and operating room, while their children usually spend less time with them due to work and family reasons, resulting in various psychological problems during their hospitalization, especially psychological stress such as anxiety and depression, and it has been proved that preoperative psychological stress is a high-risk factor that induces postoperative cognitive dysfunction in the elderly. The most common emotional response of psychological stress is anxiety. This article selected 100 patients with coronary heart disease after surgery. As a result, 48 patients had SAS scores greater than 50, and the incidence of postoperative anxiety was as high as 61%.

The article "Postoperative Cognitive Behavioral Intervention in Patients with Coronary Heart Disease Based on the Effect of Nursing Process Reengineering" was retracted in 2023. Reasons: signs of a paper mill; suspected computer-generated content; unreliable results or conclusions; lack of ethics approval or compliance.

After the patients received PCI treatment, the symptoms of the disease were relieved, and most of the patients received interventional therapy for the first time and had not experienced the process of repeated changes in the disease. Therefore, the negative emotions brought by the disease were less and the level of hope was higher. In addition, when patients learn that a good prognosis can be obtained through various ways such as drug maintenance and lifestyle changes, they have high expectations for future disease control and improvement of quality of life, making it easier for patients to obtain a higher level of hope. Different gender, education level, work status, weight classification, family monthly income per capita, smoking status, number of interventional treatments, and whether there is discomfort grouping after intervention, there is no significant difference in the level of hope of patients. It may be related to the fact that inpatient review patients have more opportunities to obtain relatively equivalent professional knowledge from medical staff's rounds, lectures, and patient-friend exchanges. Due to the development of information communication and mass media and the popularization of cardiovascular disease knowledge, although patients have different education levels and incomes, it is possible that the differences in the means and information content of obtaining disease-related information are getting smaller and smaller. Therefore, the difference in patients' understanding of the disease and the level of hope is also reduced.

The article "Postoperative Cognitive Behavioral Intervention in Patients with Coronary Heart Disease Based on the Effect of Nursing Process Reengineering" was retracted in 2023. Reasons: signs of a paper mill; suspected computer-generated content; unreliable results or conclusions; lack of ethics approval or compliance.

## 5. Conclusion

In the face of changes in the needs of patients for diagnosis and treatment services and increasingly fierce market competition, all medical institutions hope to improve their competitiveness by improving their own service quality through streamlined, flexible, and efficient organizations, catering to the needs of patients and focusing on patients. Starting to design the medical process is the ultimate goal. Therefore, the introduction of business process reengineering theory in hospital management and the reengineering of the overall hospital process have become the inevitable trend of modern hospital reform. At the same time, this article also has certain shortcomings. In terms of research content, longitudinal research can be carried out to conduct intervention research on health promotion behavior level for patients with coronary heart disease with different treatment modalities, different treatment stages, and different hope levels and coping styles and to develop targeted measures to improve the clinical prognosis and the ability to live a normal social life.

## Figures and Tables

**Figure 1:** Reengineering the preoutpatient process (pictures from Baidu picture).

**Figure 2:** Emergency node (pictures from Baidu picture).

**Figure 3:** Coronary heart disease and its treatment (pictures from Baidu picture).

**Figure 4:** Coronary heart disease electrocardiogram and blockage (pictures from Baidu picture).

**Figure 5:** Comparison of the scores of various dimensions of the quality of life in intervention group and control group in T1.

**Figure 6:** Changes of MAP and HR in the two groups of patients.

**Figure 7:** Changes of VAS score and PONV in the two groups.

**Figure 8:** Comparison of the incidence of POCD between the two groups.

**Figure 9:** Classification of self-management behavior in patients with coronary heart disease.

**Figure 10:** Changes of serum AFABP and IL-6 concentrations in each clinical subgroup before and after PCI.

**Table 1:** Patient's general information.

Index		Control group	Test group	*t*/*x*^2^/*z*	*P*
Age		63.87	64.21	−0.136	0.863
Sex	Male	26	22	0.685	0.423
	Female	11	14		

Education level	Junior high school and below	5	13	−0.321	0.815
	High school	12	10		
	Junior college	12	10		
	Bachelor degree and above	5	12		

Smoking	Yes	22	20	0.018	0.887
	No	25	25		

Drinking	Yes	22	22	0.072	0.928
	No	25	23		

Days in hospital		12.03	11.25	1.792	0.076
Doses		5.47	5.21	0.821	0.412
Pills taken		10.76	10.54	0.263	0.807

**Table 2:** Comparison of quality control standard scores between the two groups.

Time	Number	Basic nursing	Nursing operations	Specialist nursing	Ward management	Hemodialysis knowledge	Emergency medicine
Before reconstruction	25	20.76	15.87	14.76	15.23	15.87	8.43
After reconstruction	25	28.53	19.42	19.43	18.74	19.21	11.45
*t* value		10.214	4.271	4.182	4.042	4.427	3.491
*P* value		<0.001	<0.001	<0.001	<0.001	<0.001	<0.001

The article "Postoperative Cognitive Behavioral Intervention in Patients with Coronary Heart Disease Based on the Effect of Nursing Process Reengineering" was retracted in 2023. Reasons: signs of a paper mill; suspected computer-generated content; unreliable results or conclusions; lack of ethics approval or compliance.

**Table 3:** Comparison of the psychological state of the two groups of patients.

Group	Number	Somatization	Depression	Anxiety	Interpersonal sensitivity
Test group	30	1.46 ± 0.47	1.53 ± 0.45	1.47 ± 0.42	1.46 ± 0.38
Control group	30	1.77 ± 0.39	1.74 ± 0.42	1.57 ± 0.42	1.71 ± 0.29
Group	Number	Obsessive-compulsive symptoms	Hostility	Fear	Paranoid
Test group	30	1.52 ± 0.51	1.49 ± 0.27	1.32 ± 0.35	1.28 ± 0.39
Control group	30	1.74 ± 0.53	1.69 ± 0.45	1.62 ± 0.38	1.52 ± 0.51

**Table 4:** Changes in blood lipids and blood pressure in the two groups.

Group		Systolic blood pressure	Diastolic blood pressure	Total cholesterol	Triglycerides
Test group	Before joining	147.87	96.24	6.23	1.82
	After joining	125.98	74.92	5.28	1.39

Control group	Before joining	151.21	91.87	6.15	1.76
	After joining	149.64	91.25	5.98	1.69

## Data Availability

No data were used to support this study.
